# Harris Hawk Optimization: A Survey onVariants and Applications

**DOI:** 10.1155/2022/2218594

**Published:** 2022-06-27

**Authors:** B. K. Tripathy, Praveen Kumar Reddy Maddikunta, Quoc-Viet Pham, Thippa Reddy Gadekallu, Kapal Dev, Sharnil Pandya, Basem M. ElHalawany

**Affiliations:** ^1^School of Information Technology and Engineering, Vellore Institute of Technology, Vellore, India; ^2^Korean Southeast Center for the 4th Industrial Revolution Leader Education, Pusan National University, Busan 46241, Republic of Korea; ^3^Department of Institute of Intelligent Systems, University of Johannesburg, Johannesburg, South Africa; ^4^Symbiosis Institute of Technology, Symbiosis International (Deemed) University, Pune, Maharashtra, India; ^5^Faculty of Engineering at Shoubra, Benha University, Banha, Egypt

## Abstract

In this review, we intend to present a complete literature survey on the conception and variants of the recent successful optimization algorithm, Harris Hawk optimizer (HHO), along with an updated set of applications in well-established works. For this purpose, we first present an overview of HHO, including its logic of equations and mathematical model. Next, we focus on reviewing different variants of HHO from the available well-established literature. To provide readers a deep vision and foster the application of the HHO, we review the state-of-the-art improvements of HHO, focusing mainly on fuzzy HHO and a new intuitionistic fuzzy HHO algorithm. We also review the applications of HHO in enhancing machine learning operations and in tackling engineering optimization problems. This survey can cover different aspects of HHO and its future applications to provide a basis for future research in the development of swarm intelligence paths and the use of HHO for real-world problems.

## 1. Introduction

Thanks to recent advances in computing capabilities and big data analytics, artificial intelligence (AI) has been considered in various applications, ranging from natural language processing and computer vision to wireless 6G systems and medicine [1]. As a subset of AI and nature-inspired algorithms, swarm intelligence (SI) has become a hot topic over the last decade. Conceptually, SI studies the complex collective behavior of the systems that are comprised of many simple agents. More particular, these simple agents can interact with others and also with their surrounding environment. According to [2], SI has many advantages compared with the conventional optimization approaches: (1) black-box optimizer, (2) gradient-free operation, (3) ability to obtain high-quality solutions by properly balancing exploratory and exploitative features, and finally (4) ease and simplicity of implementation. These characteristics and applicability are the main reasons behind the wide use of SI approaches. Some well-known SI methods are not limited to particle swarm optimization (PSO) [3], grey wolf optimizer (GWO) [4], genetic programming (GP) [5], biogeography-based optimizer (BBO) [6], and firefly algorithm (FA) [7]. Also, SI methods have found their applications in various applications and real-world problems, such as control engineering, civil engineering, electrical engineering, image processing, wireless communications, and vertical domains (e.g., smart cities and smart grids).

Proposed by Ali Asghar Heidari in 2019, the Harris Hawks optimization (HHO) has received much interest from the research communities [8]. HHO mimics the hunting behavior of the Harris Hawks in nature, namely surprise pounce. Considered as one of the most intelligent birds in nature, Harris Hawks can simulate different chasing styles based on different scenarios and escaping prey behaviors. More specifically, four chasing strategies are developed in HHO [8], including soft besiege, hard besiege, soft besiege with progressive rapid dives, and soft besiege with progressive rapid dives. The results tested over benchmark functions and several engineering optimization problems confirm that HHO outperforms many well-known SI approaches such as PSO, GWO, GP, BBO, and FA. Moreover, the results also show that HHO achieves a good balance of exploration and exploitation, thus improving the scalability of HHO and the ability to obtain high-quality solutions.

HHO has been leveraged for many applications and engineering problems due to its optimization features and competitive performance. For example, HHO is used to solve the problem of unmanned aerial vehicle (UAV) placement and radio resource allocation in visible light communications (VLC) [9]. This work demonstrates that HHO effectively tackles the nonlinearity caused by the VLC channel modeling and solves multiple optimization variables simultaneously. The work in [10] proposes a hybrid SI method based on HHO and WOA for feature selection. To improve the production quality, a convolutional neural network (CNN) jointly with HHO is leveraged in [11], in which CNN is used to classify the control chart patterns and HHO is used to tune the parameters of the CNN model such as the number of kernels and learning rate. All the above studies show that the HHO-based method has superiority over the baseline and state-of-the-art SI methods.

According to the no-free-lunch theorem, no single algorithm can solve all the real-world problems; that is, one algorithm can perform well for a set of problems but perform poorly for the other problems [12]. Therefore, HHO has been improved by different techniques, for example, binary HHO version, evolutionary-updating structures, chaotic operations, multi-objective HHO, and hybrid HHO. As HHO is originally invented for solving continuous optimization problems, a number of studies have been conducted for binary HHO versions. For example, the work in [13] develops a hybrid SI approach by integrating HHO with the Salp swarm algorithm (SSA), which is then applied to the feature selection problem. To exploit the effectiveness of chaotic-based updates in avoiding immature convergence, the work in [14] proposed adding the chaotic local search into the original HHO to improve its performance. Another application of HHO can be found in [15], where HHO is used as a trainer of feed-forward neural networks, which is then used for load forecasting in the Queensland electric market. There is also an effort on review of a few papers on HHO in [16]. However, that paper coverage is very different, and it provides another methodology of research for conducting a review.

### 1.1. Contributions

To foster the development of the HHO and its applications, this work sets to provide an overview, recent improvements, and applications from the available literature. Motivated by this observation, we set to provide a survey on HHO, including its mathematical model, recent variants, and applications. In a nutshell, the contributions offered by our work can be summarized as follows:

- We first present the underlying inspiration and the mathematical model of the HHO optimizer. This part is to help the readers to understand the underlying principle of the HHO and how it can be applied to solve engineering optimization problems.
- We review the state-of-the-art improvements of HHO, focusing mainly on fuzzy HHO and a new intuitionistic fuzzy HHO algorithm.
- We review the applications of HHO in various disciplines such as machine learning (ML), electrical/civil/image engineering, wireless communications, and control engineering.

We note that the references reviewed in this work are obtained from high-reputed publishers such as IEEE, Elsevier, Wiley, Springer Nature, and Taylor & Francis and also well-known archival websites such as arXiv. Moreover, the following queries are used to find the references, including “Harris Hawk optimization,” “HHO,” “swarm intelligence,” “artificial intelligence,” and “metaheuristic.”

### 1.2. Paper Organization

The remaining parts of this study are organized as follows. In Section 2, we present the inspiration and mathematical models of HHO. In Section 3, we review the state-of-the-art studies on variants of HHO. Next, in Section 4, we discuss the applications of HHO in ML applications and engineering applications. Finally, we conclude this study in Section 5. The list of frequently used acronyms is summarized in Table 1.

## 2. Harris Hawk Optimization

This section presents an overview of HHO, including its inspiration and mathematical model.

### 2.1. Inspiration of HHO

HHO was proposed by Heidari et al. in 2019 to simulate the hunting behavior of the Harris Hawks [8]. In 1997, Louis Lefebvre's survey revealed that Harris Hawks are the most intelligent birds found in southern Arizona, USA [17]. The foraging behavior of Harris Hawks varies significantly from that of other birds, as Harris Hawks continue to forage with other family members of the same species. Harris Hawks use a technique called the “surprise pounce,” known as the “seven kills” approach to ambush the prey. During this attack, a few other hawks used to ambush in a number of directions and converge on the target rabbit, and the attack would be over in a matter of seconds. Harris Hawks use different hunting styles based on the escape behavior of the prey and the dynamic change in instances. For example, Hawks use switching tactics when the leader hawk dives quickly to attack the prey, and the prey is trying to escape from the leader hawk, and then, another hawk in the party team will immediately continue the chase. These switching tactics confuse the targeted prey and seek to exhaust the detected prey and increase its danger. Finally, tired prey cannot escape the hawk's team, as one of the mighty hawks slaughters the tired prey and shares it with the party members.

HHO's main inspiration is the collaborative action and hunting style of the Harris Hawk in the wildlife called the surprise pounce. The HHO mathematical model generates dynamic patterns and behaviors for the development of an optimization algorithm. The performance of the HHO optimization algorithm is evaluated by comparing it with other existing metaheuristic techniques, 29 benchmark challenges, and many real-world engineering issues. Experimental findings and comparative results have shown that the HHO algorithm delivers better results than other existing metaheuristic techniques [8, 18].

### 2.2. Mathematical Models of HHO

This section discusses the mathematical model of the HHO algorithm, which comprises an exploration phase, an exploitation phase, and a number of Harris Hawk attacking approaches. HHO is a nature-inspired algorithm that can be applied to any optimization problem. This section presents all phases of HHO, which are further explained in the following subsections.

### 2.3. Exploration Phase

In this subsection, the exploration phase of HHO is discussed. The Harris Hawks have powerful eyes that can monitor and identify prey, but sometimes the prey is not visible. During this condition, the hawks have been waiting for long hours and monitoring to identify the prey. In HHO, hawks are considered as candidate solutions, and in each iteration, the prey is considered the optimal solution. Hawks perch in specific locations and constantly monitor the surrounding environment to identify prey using two strategies, which are represented in equation (1). If *p* < 0.5, the hawks perch based on the position of the family members. If *p* ≥ 0.5, the hawks perch in a random space within the population area.

(1) $$\begin{array}{c} A\left(x+1\right)=\left\{\begin{array}{c} A_{\text{r}}\left(x\right)-a_{1}\left|A_{\text{a}}\left(x\right)-2a_{2}A\left(x\right)\right|,\;p\geq 0.5,\\ \left(A_{\text{rabbit}}\left(x\right)-A_{p}\left(x\right)\right)-a_{3},\\ \left(L_{B}+a_{4}\left(U_{B}-L_{B}\right)\right),\;p<0.5. \end{array}\right. \end{array}$$

In equation (1), where *A*(*x* + 1) denotes the position of Hacks at the next iteration. A_rabbit_(*x*) denotes the position of rabbit. *A*(*x*) denotes the current position of hawks. *a*_1_, *a*_2_, *a*_3_, *a*_4_, and *p* are random variables ranging from 0 to 1. LB and UB are the lower bound and the upper bound of random variables. *A*_*p*_(*x*) indicates the average hawk position, which is represented in the following equation, where *A*_*i*_(*x*) denotes the location of each hawk at *i*th iteration and *H* denotes the number of Hacks in the search space.

(2) $$\begin{array}{c} A_{\text{p}}\left(x\right)=\frac{1}{H}\overset{H}{\underset{i=1}{\sum }}A_{i}\left(x\right). \end{array}$$

### 2.4. Transition from Exploration to Exploitation

This subsection explains the transformation from the exploration phase to the exploitation phase, based on the energy level of the prey to escape, which is mathematically defined as follows:

(3) $$\begin{array}{c} P=2P_{0}\left(1-\frac{x}{I}\right), \end{array}$$

where *P* denotes the energy of prey to escape at iteration *x*, *I* denotes the total number of iterations, and *P*_0_ denotes the initial energy of prey. During each escape, the energy level of the prey drops dramatically. For each iteration, *P*_0_ will change the value from (−1, 1). When *P*_0_ drops down from 0 to −1, the prey is exhausted; similarly, when *P*_0_ value is increasing from 0 to 1, the prey is reinforced. When |*P*| ≥ 1, exploration took place, and when |*P*| < 1, exploitation arises.  Figure 1 represents the escaping energy behavior [8].

### 2.5. Exploitation Phase

This subsection explains the exploitation phase in which the hawks attack the targeted prey. Then, however, the prey tries to escape the attack. Based on hawk attacking behavior and escaping prey behavior, four approaches are discussed in the following subsections.

### 2.6. Soft Besiege

In HHO, soft besiege occurs when *a* ≥ 0.5 and |*P*| ≥ 0.5, and the prey has sufficient energy to escape from the attack, but cannot escape from the attack as the hawks encircle the prey and the energy of the prey gets drained. The following equations explain the mathematical behavioral model.

(4) $$\begin{array}{c} A\left(x+1\right)=\Delta A\left(x\right)-P\left|UA_{\text{rabbit}}\left(x\right)-A\left(x\right)\right|, \end{array}$$

(5) $$\begin{array}{c} \Delta A\left(x\right)=A_{\text{rabbit}}\left(x\right)-A\left(x\right). \end{array}$$

∆*A*(*x*) denotes the difference between the position vector of the rabbit and present position at xth iteration. *U* represents the rabbit's random jump strength during escape, where *U* is updated as *U* = 2 (1 − *a*_5_), and *a*_5_ is a random number ranging from [0, 1].

### 2.7. Hard Besiege

In HHO, hard besiege occurs when *a* ≥ 0.5 and |*P* | < 0.5, and the prey is exhausted and does not have enough energy. The hawks encircle the prey and perform the surprise pounce. The updated position of the hawks is shown in equation (6).  Figure 2 depicts the vectors during hard besiege.

(6) $$\begin{array}{c} A\left(x+1\right)=A_{\text{rabbit}}\left(x\right)-P\left|\Delta A\left(x\right)\right|. \end{array}$$

### 2.8. Soft Besiege with Progressive Rapid Dives

This subsection deals with soft besiege with progressive rapid dives where the prey has enough energy |*P*| ≥ 0.5 to escape the attack, but the hawk builds a soft besiege *a* < 0.5. In this step, the hawk must think intelligently and choose the best position to target the prey. The respective steps accomplish the process.

(1) Performing various moves
(2) Analyzing and thinking on a new move using equation (7)
(3) Evaluating the movement with the previous dive to the prey and realizing whether the movement is favorable or not
  (7) $$\begin{array}{c} T=A_{\text{rabbit}}\left(x\right)-P\left|UA_{\text{rabbit}}\left(x\right)-A\left(x\right)\right|. \end{array}$$
(4) If the movement is not favorable to attack the prey, a dive is selected based on a levy flight (LF) using the following equation:
  (8) $$\begin{array}{c} L=T+V\times \text{LF}\left(z\right), \end{array}$$
   where *Z* is represented as the dimension of the problem, *V* is considered as a random vector of size 1 ∗ *Z*, and LF function is calculated using the following equation:
  (9) $$\begin{array}{c} \text{LF}\left(f\right)=0.01\times \frac{m\times \psi }{\left|n\right|},\\ \psi ={\left(\frac{\xi \left(1+\chi \right)\times \text{sin}\left(\pi \chi /2\right)}{\xi \left(1+\chi /2\right)\times \chi \times 2^{\left(x-1/2\right)}}\right)}^{1/\chi }, \end{array}$$
  where *m* and *n* are random values that range between (0, 1) and *χ* is a constant that is set to 1.5. Equation (10) is used to update the positions of the hawks during the soft besiege phase.
  (10) $$\begin{array}{c} A\left(x+1\right)=\left\{\begin{array}{c} T\text{ if }F\left(T\right)<F\left(A\left(x\right)\right),\\ L\text{ if }F\left(L\right)<F\left(A\left(x\right)\right), \end{array}\right. \end{array}$$
  where *T* and *L* are acquired using equations (7) and (8), and *F* is considered to be a fitness function for the problem.  Figure 3 depicts the vectors during soft besiege with progressive rapid dives.

### 2.9. Hard Besiege with Progressive Rapid Dives

This subsection deals with hard besiege with progressive rapid dives when |*P*| < 0.5 and *a* < 0.5 where the prey does not have enough energy to escape the attack and hawk builds a hard besiege to catch and kill the prey. In this phase, the prey's condition is similar to that of the soft besiege, but the hawks intend to minimize the distance between their locations towards escaping prey. The equation explains the hard besiege condition.

(11) $$\begin{array}{c} A\left(x+1\right)=\left\{\begin{array}{c} T\text{ if }F\left(x\right)<F\left(A\left(x\right)\right),\\ L\text{ if }F\left(x\right)<F\left(A\left(x\right)\right), \end{array}\right. \end{array}$$

where *T* and *L* are derived using the following equations.

(12) $$\begin{array}{c} T=A_{\text{rabbit}}\left(x\right)-P\left|UA_{\text{rabbit}}\left(x\right)-A_{p}\left(x\right)\right|, \end{array}$$

(13) $$\begin{array}{c} L=T+V\times LF\left(z\right). \end{array}$$

Figures 4 and 5 depict vectors during hard besiege with progressive rapid dives in 2D and 3D space. Algorithm 1 explains pseudocode for HHO.

## 3. Recent Variants of HHO

This section discusses various HHO variants that are used in a variety of engineering and ML applications, as shown in Tables 2–4. We discussed the fuzzy HHO in this section and proposed a new intuitionistic fuzzy HHO algorithm that is significantly different from other existing papers [16].

### 3.1. Fuzzy Harris Hawk Algorithm

Fuzzy sets [48] were introduced as an extension of crisp sets to take care of graded membership of objects in a class, which are more general and natural. This has led to the extension of crisp concepts to fuzzy concepts. Fuzzy logic (FL), in the generalized sense, is synonymous with fuzzy sets. One of the crucial components of FL is the fuzzy inference system (FIS).

A FIS has five functional blocks, a rule base that contains several fuzzy If… then rules. In addition, this database defines the membership functions of fuzzy sets used in fuzzy rules. This decision-making unit operates on the rules, a fuzzification interface unit that converts crisp quantities into fuzzy quantities and a defuzzification interface unit that converts the fuzzy quantities into crisp quantities. FIS is the most critical tool in fuzzy set theory, and in literature, we find two crucial FIS: the Mamdani FIS proposed in 1975 [49] and the Sugeno FIS proposed in 1985 [50]. Of these, Mamdani FIS is the popular one and finds a greater acceptance. However, both approaches have certain advantages and disadvantages. The significant differences are in the output membership functions and the consequents of the fuzzy rules used. As far as the functionality of a FIS is concerned, if the input is crisp, it is fuzzified in the fuzzification unit using one of the various fuzzification techniques. Fuzzification is the process of decomposing a system input and/or output into one or more fuzzy sets. Many types of curves and tables can be used, but triangular- or trapezoidal-shaped membership functions are the most common, since they are easier to represent in embedded controllers. A set of fuzzy if-then rules are determined. The rule strengths are obtained by combining the fuzzified inputs. The output membership function is combined with rule strength to obtain the consequent. An output distribution is obtained by combining all the consequents. The defuzzification unit is used to get a defuzzified output distribution.

The two parameters involved in the HHO algorithm are the energy of the prey *E* and the uniform random number parameter *q*, which determines the hawk's position the next time. The general tendency to fuzzify any algorithm is to fuzzify its parameters. Following the same approach in developing the fuzzy HHO (FHHO), the parameters *q* and *E* have been fuzzified by the researchers and were introduced in [51]. To achieve this, the Mamdani FIS model is used in this study. In many cases, we find the inputs in the crisp form only. However, the beauty of fuzzy logic is the way it turns common sense, and linguistic descriptions, into a computer-controlled system. Hence, the crisp inputs are transformed into fuzzy forms and then transformed into fuzzy form at the first stage of FIS.

Figure 6(a) shows a system of fuzzy sets for an input with trapezoidal and triangular membership functions. Each fuzzy set spans a region of input (or output) values graphed against membership. Any particular input is interpreted from this fuzzy set, and a degree of membership is obtained. The membership functions should overlap, to allow smooth mapping of the system. The process of fuzzification allows the system inputs and outputs to be expressed in linguistic terms to allow rules to be applied in a simple manner to express a complex system. In Figure 6(a), the fuzzy variable DF can take four linguistic values, e.g., small, medium, big, and very big. The linguistic values small and very big are represented by trapezoidal-shaped membership functions, whereas the linguistic values medium and big are represented by triangular-shaped membership functions. The inputs provided to Mamdani FIS to generate these two parameters *q* and *E* are the input variables df and NU, where df represents the quality of the best solution at the end of a searching iteration and NU represents the number of iterations with the unchanged best solution.

(14) $$\begin{array}{c} \text{df}=\text{CP}\left(t\right)-\bar{\text{CP}}. \end{array}$$

The coverage percentage of the observed area determines the quality of the solution. So, we have the coverage percentage at the iteration number *t,* which is denoted by CP(*t*), and the arithmetic mean of the obtained covered percentages is represented by $\bar{\text{CP}}$. NU is also normalized to NU and is given by the following expression:

(15) $$\begin{array}{c} \text{NU}=\frac{\text{NU}-{\text{NU}}^{\min}}{{\text{NU}}^{\max}-{\text{NU}}^{\min}}, \end{array}$$

where *NU*^max^ and *NU*^min^ are the maximum and minimum values of NU, respectively. The inputs df and NU are fuzzified using the fuzzification process. df and NU are fuzzy variables, with each one taking the values from the domain of fuzzy granules medium, big, very big, and small (Figure 6). Together, these two variables can take 16 values, and accordingly, 16 rules are framed. The antecedents contain these 16 values, and the consequent provides 16 pairs of values for the fuzzy variables energy and *q*. Energy takes 8 values (here P denotes positive and N denotes negative) leading to NVB, NB, NM, NS, PS, PM, PB, and PVB and *q* takes values small, medium, big, and very big. There were 16 fuzzy rules in the rule base; e.g., DF is medium and NU is small and then energy is PM and *q* is medium.

3D sensors were reallocated in FHHO to supervise cardiomyopathy. The candidate solutions of the n-hawks in the vector form of candidates are {*x*_*n*_, *y*_*n*_, *z*_*n*_} in the observed area. So, the dimension of the hawks will be three times the number of sensors required.

Two validation experiments were conducted to evaluate the performance of the FHHO algorithm with different scenarios. Three different scenarios were formulated, and the performance was compared with several other AI algorithms with an iteration of 150 and the number of search agents being 10. It has been observed that FHHO reaches the best coverage value. This is concerning 30 runs. In another experiment, another constraint is added so that the search space reduces in size leading to difficulty in obtaining the best solution. In this case, the number of iterations is fixed at 200. Keeping with the additional constraint, the coverage rate of FHHO was found to be higher. Here also several cases are considered. Wilcoxon signed-rank statistical analysis [52] shows that in comparison with other algorithms, FHHO has a higher coverage percentage. Also, violations of constraint for FHHO are significantly small as the tie's values are minimal.

### 3.2. Proposed Variants of HHO

#### 3.2.1. Intuitionistic Fuzzy HHO Algorithm

Exact membership functions are used in FIS. In the systems where insufficient information about imprecise concepts is provided, FIS may not be useful. Intuitionistic fuzzy sets (IFSs) provide additional information about imprecise concepts. In the case of fuzzy sets, the membership functions and nonmembership functions are one's complement of each other. Nevertheless, by relaxing this constraint, such as their sum lies in [0, 1], we get the IFS, which has an additional parameter called the hesitation. IFIS has been proposed in many ways. However, they have the problem of overfitting and being unable to deal with complex systems, So, an IFIS that comes over these difficulties has been proposed in [53] by generating the if-then rules through the fuzzy association mining algorithm. They have used the Takagi-Sugeno type of FIS. In fact, the two types of FISs differ in their ways of generating the outputs. The different formulation of outputs leads to different if … then rule formulation. The if … then rules are automatically extracted from the input data, and logical connectives AND, OR, and NOT are used in these rules in framing implications and aggregations of these rules. The number of if … then rules can also be optimized. In the Takagi-Sugeno, FIS has higher computational effectiveness as defuzzification is not required.

Let *U* be a non-empty set. Then, an IFS A over U is defined as the set of tuples {(*x*, *μ*_*A*_(*x*), *v*_*A*_(*x*))|*x* ∈ *U*}.

Where *μ*_*A*_, *v*_*A*_ : *U*⟶[0,1] such that 0 ≤ *μ*_*A*_(*x*)+*v*_*A*_(*x*) ≤ 1,  ∀ *x* ∈ *U*. Here, *π*_*A*_(*x*)=1 − *μ*_*A*_(*x*) − *v*_*A*_(*x*) is called the hesitation margin. An IFS A is a fuzzy set if and only if *π*_*A*_(*x*)=0,  ∀ *x* ∈ *U*. The *π*_*A*_(*x*) is called the IF indices. Larger *π*_*A*_(*x*) values lead to a higher hesitation margin by the decision-maker. Best (or worst) final results are determined by these indices, which are finally in an optimal decision. With the above notations, if *y*^*η*^ is the output of an IF system then with *y*^*μ*^ and *y*^*v*^ being the outputs of the two FISs *F*^*μ*^ and *F*^*v*^ of the membership and nonmembership functions, we have the relation as follows:

(16) $$\begin{array}{c} y^{n}=\left(1-\pi_{A}\left(x\right)\right)y^{\mu t}+\pi_{A}\left(x\right)y^{\nu }. \end{array}$$

This is the fundamental equation in designing the Takagi-Sugeno type IFIS.

#### 3.2.2. First Version of IFIS

Two FISs FIS^*μ*^ and FIS^*v*^ are formed using the membership function *μ*_*A*_ and the nonmembership function *v*_*A*_. This is called IFIS with composition defuzzification [53, 54]. Here, *x*_1_, *x*_2_,…*x*_*m*_ are input variables and one output variable *y*^*η*^.

### 3.3. IFHHO Algorithm (Proposed)

We may note that the efficiency of the IFIS over the FIS is established in [55] by taking the real-life application of genetic tuning for predicting financial performance, plant monitoring in [56], and air quality modeling in [57].

## 4. Applications of HHO

This section discusses various ways in which HHO can be used in ML and engineering applications. Also, the recent state of the art on applications of HHO and its variants in several applications is discussed. The summary of these applications is pictorially summarized in Figure 7.

### 4.1. Machine Learning Applications

Lefebvre et al. [17] observed the feeding behaviors of different species based on the avian “IQ.” In [17, 58, 59], he listed hawks as one of the most intelligent birds. The Parabuteo unicinctus (Harris Hawk) belongs to the same hawk species listed in the intelligent bird category. The Harris Hawk is mainly found in Arizona, USA [60]. The Harris Hawk follows the “surprise pounce” strategy to capture its prey, suggesting that several hawks from different directions attack cooperatively and converge simultaneously to the detected prey (rabbit). The chasing styles of Harris Hawk may adapt to the dynamic nature and prey's escape pattern. The Harris Hawk can also perform a switching strategy, suggesting that if the leader (best hawk) loses its way to the prey while performing a quick dive, a member of the same hawk fleet will continue the chase. This tactic is helpful as it confuses the prey and might exhaust the prey. Inspired by its attack tactics, the Harris Hawk optimization (HHO) method was proposed [8]. The HHO follows mainly two stages to hunt its prey, i.e., exploration and exploitation. The exploration phase is related to discovering its prey, and the exploitation is to decide whether hard or soft besiege should be applied. The hard besiege is applied when the prey is fatigued, and the hawk can perform surprise pounce, while the soft besiege is used when the prey possesses adequate energy to escape. The transition stage models the energy of its prey. We consolidate a brief review of existing works using the HHO method.

### 4.2. Harris Hawk Optimization for Artificial Neural Networks

HHO method is categorized as one of the metaheuristic approaches, which are extensively used to optimize the hyperparameters of ML algorithms such as artificial neural networks (ANNs), support vector machines (SVMs), and so forth [61, 62]. Some of the works summarizing the use of HHO for ANN parameter optimization are elaborated. Sammen et al. [63] proposed the use of HHO for optimizing the weights in ANN. The method was applied to predict the scour depth for ski jumping. They mainly computed the energy parameter and jumped strength for HHO and weight optimization for ANN. Their analysis showed that the weights optimized through HHO yield the lowest mean absolute percentage error, mean absolute error, and root-mean-square error compared with ANN without metaheuristic, genetic algorithms, and particle swarm optimization. Furthermore, they also showed that HHO achieves the best correlation coefficient and Willmott index values for scour depth prediction compared with the techniques mentioned above. Similarly, Essa et al. [64] used HHO to optimize ANN weights for the prediction of active and solar stills. Their experimental results revealed that HHO-optimized ANN can provide 53.21% increased productivity concerning active still in comparison with traditional ANN and SVM classifiers. The same conclusion was drawn by Moayedi et al. [37] when using HHO-optimized ANN for soil conditions. They concluded that the HHO-optimized ANN can decrease the mean absolute error by 11.32% and 4.12% for seen and unseen soil conditions compared with traditional ANNs. Moayedi et al. in [29, 65, 66] explored the use of HHO with ANN for predicting landslide vulnerability, bearing ability over soil footing, and slope stability, respectively. The results revealed that the HHO improves the predictive performance in both studies compared with the conventional ANN method. Wei et al. [20] improved the HHO's performance using the Gaussian barebone strategy to optimize kernel extreme learning machines for the prediction of entrepreneurial intention. The Gaussian barebone allows the population to opt for the directions, which leads to faster convergence. Their results showed better and promising results in terms of specificity, sensitivity, accuracy, and Matthews correlation coefficient.

### 4.3. Clustering and Segmentation

There are a few studies that specifically use the HHO method for the clustering and segmentation process.

Pham et al. [67] proposed the use of HHO for joint power allocation and UAV placement problems. Their study used HHO in conjunction with an efficient user clustering strategy to allocate the power resources for UAV-assisted systems. The comparison was carried out with orthogonal multiple access, non-orthogonal multiple access with visible light communication, non-orthogonal multiple access without pairing, and random user clustering. Experimental results show that the HHO-based clustering outperforms the techniques mentioned earlier for power allocation and UAV placement problems.

Singh [21] used the HHO with chaotic sequences for the application of data clustering. The clustering performance was compared with various ML algorithms on 12 benchmark datasets. It was revealed that the HHO performs better on the majority of the benchmark datasets in terms of statistical tests and performance analysis. Jia et al. [22] employed mutation operator and dynamic control strategy to balance the exploitation and exploration phases in the HHO method. The modified HHO was used to perform segmentation on satellite and oil pollution images. The results were compared with several thresholding methods in terms of Otsu between-class variance, Tsallis entropy, and Kapur's entropy. The results revealed that the HHO-based approach outperforms the thresholding techniques for the specified segmentation task.

Rodrıguez-Esparza et al. [68] used the minimum cross-entropy function to optimize HHO for multilevel image segmentation task. The performance of HHO-based method was compared with fuzzy IterAg and K-means clustering. It was shown that the HHO performed better on the said segmentation task in terms of peak signal-to-noise ratio, feature similarity, and structure similarity. Bao et al. [23] proposed the hybridization of the HHO method by making two equal subpopulations from a complete one and train both the subpopulation using HHO and differential evolution, accordingly. The hybridized HHO was then used to perform multilevel image segmentation on 10 benchmark datasets. Compared with super-pixel segmentation approaches, the results revealed that hybridized HHO performs better in terms of feature similarity and structure similarity, respectively. Wunnava et al. [24] proposed an adaptive HHO method by clipping the range and constraining the escape energy. Furthermore, they allowed the method to decide whether to opt for average fitness value and approach a tall tree or roost and other hawks in the family. The adaptive HHO was used for multilevel image segmentation on the Berkeley segmentation dataset and was compared with well-known segmentation methods. Experimental results showed that the adaptive HHO achieved state-of-the-art segmentation performance.

### 4.4. Feature Selection

HHO has been used extensively for the feature selection process to optimize the parameters for classification methods [69, 70]. Ismael et al. [25] proposed to improve the HHO method by employing an opposition-based learning approach (OBL). The OBL generates a solution for meta-heuristic algorithms through an adversarial learning approach. The OBL-HHO was applied to select the informative features from the feature space in conjunction with support vector regression. Their experimental results proved that OBL-HHO achieved better results in comparison with cross-validation and grid search methods.

Sihwail et al. [26] proposed an improved HHO using elite opposition-based learning (EOBL). The EOBL stacks upon OBL by selecting the fittest individual that would direct the population towards global minimum. The improved HHO was used to select informative features from the feature space and was compared to well-known optimizers such as slime mould, butterfly optimization, whale optimization, ant lion optimization, and grasshopper optimization. Experimental results revealed that the improved HHO performed better in terms of fitness value, accuracy, and feature selection compared with the techniques mentioned earlier.

Abdel-Basset et al. [27] modified the HHO method using simulated annealing and bitwise operations and termed it as HHOBSA. The bitwise operations help HHO improve the feature selection process, whereas the simulated annealing helps HHO find the global minimum. It was revealed in their experimental results that HHOBSA performed better on 19 artificial and 24 standard datasets in comparison with the classical HHO.

Elgamal et al. [28] also used simulated annealing to improve HHO. In addition, they also introduced chaotic maps instead of random variables to achieve global optimum. The chaotic HHO was used for selecting the most informative features to train using K-nearest neighbor for the classification task. The results reveal that the chaotic HHO achieved the best accuracy against several optimization algorithms.

Zhang et al. [13] improved the HHO algorithm by adding the Salp swarm optimization, which adjusts the populations and uses greedy selection to update the agent. The Salp swarm optimization is also used to maintain a balance between the exploitation and exploration phases. The improved HHO is applied in a binary tree strategy to select the informative features. Their proposed method was used in conjunction with K-nearest neighbor and is compared with classical swarm-based approaches. Experimental results show that their improved HHO performs better on the optimization functions and classification tasks. Thaher and Arman [71] also used binary tree-like structure with HHO to select the informative features. They trained the selected features with three classification algorithms: linear discriminant analysis, decision trees, and K-nearest neighbor on SFP classification datasets. Their results show that the selected features from HHO, when trained with linear discriminant analysis, achieved the best accuracy. Houssein et al. [72] proposed the use of HHO to find the chemical compound activities and descriptor selection followed by the training using SVM and K-nearest neighbor, accordingly. The experiments were carried out to compare the HHO-SVM and HHO-K-nearest neighbor-based methods with the classical optimization algorithms on QSAR biodegradation and monoamine oxidase datasets. The HHO-SVM provides superior results on both datasets in comparison with all other algorithms.

### 4.5. Support Vector Machines and Support Vector Regression

Like the studies with ANN, the HHO method has been used to perform parameter optimization of SVM and support vector regression techniques. For example, Tikhamarine et al. [65] presented a rainfall-runoff prediction technique using least-squares SVM, ANN, and multiple linear regression optimized through the HHO method. Their study performed a detailed comparative analysis and concluded that the least-squares SVM optimized through HHO achieves the best precision values compared with the other classification algorithms. Fu et al. [29] suggested that the control formula in HHO is linear, suggesting that the optimization at the start of the process focuses more on exploration, whereas the focus diverts to the exploitation at a later stage. They proposed an improved hybrid differential evolution HHO by proposing nonlinear control formula that balances the exploitation and the exploration throughout the convergence process. They used the improved version of HHO to optimize phase space reconstruction and kernel extreme learning machine parameters for wind speed forecasting and showed that the improved version achieves better results than the HHO optimized classifiers.

Malik et al. [66] performed a comparative analysis for water stream flow prediction by employing support vector regression optimized through multiple metaheuristic approaches that include Bayesian optimization, particle swarm optimization, HHO, spotted hyena optimizer, multi-verse optimizer, and ant lion optimization. The methods were evaluated in terms of the Willmott index, correlation coefficient, scatter index, and root-mean-square error. They concluded that the support vector regression optimized through HHO yields the best results among all optimization techniques. Shao et al. [30] added periodic mutations for enhancing swarm diversity in the basic HHO method and termed it as vibrational HHO. They used the vibrational HHO to optimize SVM parameters for roll-bearing fault diagnosis. The vibrational HHO outperformed 23 benchmark functions with a faster convergence rate.

Furthermore, the HHO method has been used for various other tasks such as structural design optimization of vehicle components [73], manufacturing optimization problems [74], polluted distribution [75], heat sink design for micro-channel [76], photovoltaic cell optimization [14], and many more.

### 4.6. Engineering Applications, Electrical Engineering and Renewable Energy

Due to the numerous installations of photovoltaic (PV) power plants, the accurate modeling of PV modules is the need of the hour. Qais [77] proposed a three-diode photovoltaic (TDPV) model for the accurate modeling of photovoltaic losses. The authors have employed the HHO algorithm to extract the unknown parameters of the TTDV model. The authors have utilized datasheet values of PV modules that the industrialists provide to identify 4 of 9 unknown parameters of the TDPV model, and the HHO algorithm is employed to extract the remaining five parameters. The experimental results proved that the proposed HHO-based TDPV model performed better than the existing models. In a similar work, Hussein [31] presented a boosted HHO algorithm to estimate the parameters efficiently for a single-diode PV model. The proposed boosted HHO algorithm enhances the HHO algorithm by integrating it with the exploratory phase of the flower pollination algorithm and mutation step of differential evolution. Chen [14] proposed the HHO-based model for the estimation of solar cell models for single diode, double diode, and PV modules. The proposed HHO-based model is based on opposition-based exploratory strategy and chaotic drifts to identify the optimal agents and unknown PV model parameters.

Mansoor et al. [78] proposed an MMPT controller based on HHO to track the power effectively in solar-powered PV systems in all the weather conditions. The HHO algorithm is proven to achieve faster convergence and track maximum power point. Proton exchange membrane fuel cell (PEMFC) is one of the most importantly environmentally friendly energy sources. Mossa et al. [79] have used a hybrid of atom search optimization and HHO to extract the PEMFC's unknown parameters. The proposed hybrid algorithm is tested on 3 different PEMFC stacks, 250W stack, 500W SR-12 PEM stack, and BCS 500-W PEM stack, respectively, in several operating conditions. In a similar work, Menesy et al. [35] applied a chaotic HHO algorithm to accurately estimate the proton exchange membrane fuel cell's operating parameters that can mimic and simulate its electrical performance. The authors have used an enhanced HHO with 10 chaotic functions to avoid local optima trapping of conventional HHO.

Liu et al. [32] proposed an improved HHO for simulating an efficient PV system and to extract the unknown parameters. To prevent the HHO from falling into local optima, the authors have used a crisscross optimizer and Nelder–Mead simplex algorithm to improve individuals' searching capabilities for achieving a faster convergence rate. In a similar work, Yousri et al. [34] have proposed a modified HHO to relieve the PV systems from the issue of mismatch power loss problems resulting due to the phenomenon of partial shading. The modified HHO provides the optimal reconfiguration pattern for the switching matrix for maximizing the power generated from the array.

The safe operation and rational dispatching of a power system depend on the accurate prediction of wind speed. Fu et al. [33] have employed a hybrid of HHO and GWO for optimizing the parameters of phase space reconstruction and kernel-based extreme learning machine algorithms to predict the wind speeds accurately. The end users can communicate with the operators of the grid through a demand-side management program. This program can help the customers to take the assistance of grid operators to reduce the power consumption of the utilities during peak hours by smartly managing the load. Mouassa et al. [80] employed HHO to schedule energy in smart homes. Abdel Aleem et al. [75] have employed HHO to reduce the harmonic overloading levels of components based on the frequency with optimal planning of C-type harmonic filter, which is resonance free in a non-sinusoidal distribution system. Selim et al. [36] have employed HHO and multi-objective HHO to find the location of distribution generation optimally in a radial distribution system to minimize the voltage deviation and total active power loss and also to increase the voltage stability index under several operational constraints.

### 4.7. Civil Engineering

Many researchers have used the HHO algorithm to solve some of the critical research problems in the civil engineering (CE) domain, such as predicting the stability of the soil slopes accurately, optimizing structural design problems, air pollutant forecasting, and predicting the blast-induced ground vibration. The rest of this subsection presents recent research works that solved several CE problems.

One of the essential parameters to estimate the settlement of soil layers in CE applications is soil compression coefficient (SCC). Moayedi et al. [37] have proposed a hybrid of HHO and grasshopper optimization algorithm (GOA) to optimize the artificial neural network (ANN) for predicting SCC. The authors have used the ensemble of GOA and HHO to tune and find the optimal parameters of the ANN. The dataset is then trained and tested by the proposed model to predict SSC. To further improve the ANN-GOA prediction model, the authors have proposed a hybrid GOA-HHO algorithm for the prediction of SSC. Another challenging issue in CE is predicting the stability of the soil slopes (SSs). Moayedi et al. [81] proposed the HHO-based convolutional multilayer perceptron model to predict safety factor in constructions with rigid foundations based on SS conditioning factors. The HHO algorithm is used in this work to adjust the computational weights of the SS abovementioned factors.

Guardrail systems are designed to absorb the energy generated by vehicles driven on the roads to increase the safety of motorways. Enes Kurtulus et al. [38] proposed a hybrid HHO-simulated annealing (HHOSA) for optimizing real-world structural design problems. The HHOSA algorithm is used in this work to optimize the design parameters of highway guardrail systems.

Due to the increase in industrialization and motor vehicles, air pollution is increasing daily in several parts of the globe rapidly. Air pollution is affecting the environment badly and endangering all kinds of species. Global warming is also the result of an increase in air pollution. Even though several researchers have conducted several studies, they had significant deficiencies such as insufficient initial parameters and neglecting the significance of predictive stability, which affected the performance of air pollution forecast models. Du et al. [19] proposed the HHO-based extreme learning ML model to overcome the deficiencies of existing models.

Blasting and drilling are the conventional methods for fragmentation of the rock mass in mines as they are efficient and cheap. However, the vibration generated by the blasts can damage the surrounding structures and rock. To control the damage induced by blasting, an efficient prediction model must be designed for controlled blasting in mines. Yu et al. [82] have proposed the HHO-based random forest algorithm to predict the vibration induced by the blast. HHO is used for tuning the parameters of the random forest algorithm. To increase the samples by randomly changing the values of the attributes, the authors have used the Monte Carlo simulation method.

A spillway, which is a structure that regulates discharge flowing from massive hydraulic structures such as dams, plays a pivotal role in the safety of the dams. A spillway also dissipates the extra energy of water with the help of still basins. However, the high flow velocity on the spillway may lead to a serious problem known as bed scouring, resulting in spillway failure and soil erosion. Sammen et al. [63] have proposed a hybrid ANN-HHO model to predict the ski jump spillway's scour depth downstream. The HHO algorithm is used in this work to tune the parameters of the ANN. In a similar work, Khalifeh et al. [83] have proposed a model based on HHO to optimize the water distribution network in Homashahr, Iran, from September 30, 2018, to October 30, 2019. In this article, the researchers have integrated HHO with EPANETE 2, a water distribution network analyzing software. The EPANET 2 software analyzes the velocity of flow for every pipe and the pressure of every node. The diameter of the pipes is the main optimization parameter used in this work. The main objective is to design optimal water distribution systems. The HHO algorithm is used in this work to choose the optimal parameters.

The effects of several uncertainties, such as load, dimension, and material properties, are to be considered in the design and analyzing the risk of structures in CE. Prediction of failure probability in reliability problems with high dimensions is a significant research problem. The first-order reliability method (FORM) is a popular method used in CE for reliability analysis. However, FORM suffers from divergence or convergence issues when dealing with high dimensions with nonlinear limit state function. To address the issue of high dimensionality, Zhong et al. [39] presented an improved FORM based on the HHO algorithm. The HHO algorithm is used to choose optimal algorithmic parameters for FORM.

### 4.8. Image Processing

Several nature-inspired computing algorithms including HHO have been efficiently used by researchers in solving many problems in image processing, such as digital mammogram segmentation, image thresholding, and removing the noise from the images [84–86]. The recent state-of-the-art works by researchers on applications of HHO in image processing are discussed in the remainder of this subsection. One of the crucial phases in image processing is segmentation, as it simplifies image representation through which it facilitates the analysis. Rodrıguez-Esparza et al. [40] have proposed a HHO-based methodology for multilevel segmentation of images. Minimum cross-entropy thresholding (MCET) is used as a fitness function for HHO in this work. To find the optimal configuration of thresholds for image processing, the HHO algorithm is used in this work.

One of the drawbacks of the traditional HHO algorithm is its limited exploration ability, as it gets completely exhausted when the escape energy is zero. Wunnava et al. [42] have proposed a novel differential evolutionary adaptive HHO (DEAHHO) to address the issue mentioned above. The authors have modified the exploration phase of HHO within the range of [2,0] to limit the escape energy. The authors have also updated the HHO by making the Harris Hawk adaptive to decide when it has to move to a random tall tree or when it has to do perching. Also, to improve the exploration ability of HHO, the authors have used the differential evolutionary concept. Multilevel image thresholding methods based on 1-*D* histograms have been using Masi entropic function recently. However, the problem with the current approaches is the missing of contextual information in the 1D formulation. To address this issue, a novel 2D practical Masi entropy function is proposed by the authors. DEAHHO has been applied in the proposed 2D practical Masi entropy-based multilevel image thresholding while segmenting the images. To validate the DEAHHO method, the authors have considered 23 popularly used benchmark test functions. For experimentation purposes, 500 images are obtained from the renowned Berkeley segmentation dataset. PSNR, FSI, and SSI metrics are used to evaluate the performance of the proposed method. The proposed method yielded better results when compared to other state-of-the-art algorithms. In a similar work, Wunnava et al. [24] have used the abovementioned updated HHO along with an improved 2D grey gradient method to preserve the edge information of images with high magnitude. The same dataset used by [42] is used in this work to evaluate the proposed method. Designing an efficient automatic brain tumor classification model is the need of the hour as the precision of existing classification models is not satisfactory. Rammurthy and Mahesh [41] proposed a hybrid WOA-HHO (WHHO)-based deep CNN model [87] for classifying brain tumor using MRI images. In this work, rough set theory and cellular automata are used to perform the segmentation of MRI images. The features extracted from the MRI images are variance, mean, local optical-oriented pattern, kurtosis, and tumor size. To tune the parameters of the deep CNN model, the WHHO optimization algorithm is used. The datasets used to train the proposed model are simulated BRATS dataset (dataset 3) and BRATS dataset (dataset 4). The metrics used to evaluate the proposed model are accuracy, specificity, and sensitivity.

HHO algorithm may be struck due to local optima problem and may suffer immature convergence during the exploitation and exploration phases. To address these issues in HHO, Abd Elaziz et al. have proposed [43] a hybrid HHO-SSA optimization algorithm for multilevel image segmentation problems. The proposed model addresses the global optimization problem and also helps in finding optimal threshold values. In the proposed work, the first initial set of solutions is generated. Later, these solutions are divided into two halves. The exploitative and exploratory phases of HHO will be applied to the first half of the solutions, whereas in the second half, the searching stages of SSA will be applied. Later, the optimum solutions from these halves are chosen to continue the rest of the iterative process. 11 natural gray-scale images and IEEE CEC 2005 benchmark functions are used to perform experiments. The measures used to evaluate the proposed method are average fitness value, worst fitness value, best fitness value, and the standard deviation. The experimentation results proved that the hybrid HHO-SSA performs better than the individual algorithms and several other popular algorithms. Removal of noise from images is essential during image processing as the further procedure is not possible with noisy images. Researchers have recently attempted to improve the quantitative and qualitative results by removing the noise from the images. However, the attempts from researchers could not preserve the image quality after the application of de-noising methods. Golilarz et al. [88] used the HHO algorithm for optimal image de-noising to tune the parameters of the thresholding functions. In this work, HHO is used to obtain the best-thresholded values for wavelet coefficients before applying the inverse wavelet transforms in the first stage. In the next stage, the authors have presented an improved adaptive generalized Gaussian distribution threshold algorithm that is a data-driven function that has an adaptive threshold value. The proposed function can fit all kinds of images without the usage of a shape tuning parameter. The authors have used six satellite images for experimentation. The results proved that the proposed model achieved better accuracy and less time to process the data when compared to traditional models. In a similar work, Golilarz et al. [44] proposed a hybrid multi-population differential evolution-HHO (CMDHHO) algorithm for optimizing de-noising in satellite images in the wavelet domain. The experimental results have proved that the proposed CMDHHO algorithm yielded better quantitative and qualitative results when compared to several other optimization algorithms and thresholding neural network approaches. CMDHHO also improved the processing time and also proved to be computationally efficient. PSNR and mean SSI are the attributes used to evaluate the performance of the de-noising algorithms considered in this work.

Implementation of multilevel thresholding for color images is time-consuming and complex as the information that has to be processed is high, and also, the number of thresholds is more for color images. Bao et al. [23] have proposed a hybrid algorithm based on HHO for image segmentation of color images. The proposed hybrid model is a combination of HHO and differential evolution (DE). This hybrid algorithm, HHO-DE, extracts optimal features from images for the segmentation of color images. Kapur's entropy and Otsu's method are used as fitness functions to find the threshold values of segmentation. The proposed model divides the entire population into two equal parts assigned to DE and HHO algorithms. During the iterative process, both HHO and DE will update each subpopulation's position simultaneously. The proposed model is implemented on 10 benchmark images. The proposed model is then compared with 7 state-of-the-art methods. For evaluating the performance of the algorithms, 5 measures, FSI, SSI, PSNR, standard deviation, and average fitness values, are used in this work. The comparative analysis proves the superiority of the proposed HHO-DE algorithm. In a similar work, Jia et al. [89] proposed the application of the HHO algorithm for tuning of parameters by pulse coupled neural network (PCNN) method for the segmentation of medical images. The proposed HHO-PCCN method reduced the number of parameters of PCNN without affecting the effect of segmentation. In a similar work, Jia et al. [22] proposed a novel dynamic HHO algorithm with a mutation mechanism for segmentation of satellite images. Compared with the traditional HHO algorithm, the proposed dynamic HHO with a mutation mechanism can overcome the problem of falling into local optimum, increasing the searching capacity. Landslides are one of the most devastating environmental threats that can cause substantial financial and physical damage worldwide. Predicting the landslides reliably can save lives and also reduce damages to property. Bui et al. [90] have used the HHO-based ANN to analyze landslide susceptibility in Western Iran. In addition, HHO is used to tune the parameters of ANN.

### 4.9. Mechanical Engineering

Essa et al. [64] have proposed an HHO-ANN model to predict the productivity of active solar still, which is used to extract fresh drinkable water from water with a high concentration of salt (briny water). The HHO algorithm is used in this work to select optimal parameters of ANN. The experiments were conducted at the Faculty of Engineering, Kafrelsheikh University, Kafrelsheikh. Song et al. [45] have proposed a hybrid cuckoo search-HHO algorithm to solve three classical mechanical engineering problems: five-stage cantilever beam design problem, welded beam design problem, and tension/compression spring design problem. The cuckoo search-based HHO algorithm is used to optimize the parameters in the engineering abovementioned problems. The proposed algorithms achieved better results when compared with other metaheuristic algorithms.

Friction stir welding has proved to be efficient in welding materials when compared to traditional fusion welding methods. Shehabeldeen et al. [91] have proposed an adaptive neuro-fuzzy inference system integrated model integrated with HHO to predict the mechanical properties of friction stir welding. The HHO algorithm is used to find the optimal parameters of the adaptive neuro-fuzzy inference system and find optimal conditions of the friction stir welding process. Micro-channel heat sinks are one of the popular methods to remove heat and cool the integrated circuits in electronic devices. Entropy generation is a negative factor for micro-channel heat sink systems. Abbasi et al. [76] applied HHO optimization to minimize the entropy generation in micro-channel heat sinks.

The grinding process is a basic shaping method that is used to sharpen weapons and piercing cutting. It is used in the manufacturing of various tools. Providing optimal surface quality is the aim of the grinding process. The optimization of production rate and production cost is crucial in the grinding process to ensure surface quality. Yıldız et al. [74] have used HHO, GOA, and multi-verse optimization algorithm (MVO) to optimize the processing parameters in grinding operations. Jouhari et al. [46] proposed a hybrid HHO-SSA algorithm to address scheduling problems in unrelated parallel machines. In this study, SSA is employed to enhance the performance of HHO by acting as a local search for HHO. As a result, the proposed hybrid algorithm resulted in improved performance and reduced computational time.

To solve shape optimization problems in manufacturing industry, Yıldız et al. [74] employed HHO, SSA, GAO, and dragonfly algorithm. In this work, HHO, SSA, GAO, and dragonfly algorithms are applied for optimizing the shape of the vehicle brake pedal. Singh [47] proposed a hybrid HHO-WOA-based ANN to predict emission properties of a single-cylinder direct injection diesel engine. The proposed hybrid HHO-WOA algorithm optimized ANN to predict the values of several parameters such as hydrocarbon, brake thermal efficiency, carbon monoxide, and carbon dioxide.

### 4.10. Wireless Communications and Internet of Things

Fiber wireless (FiWi) integrates wireless and optical networks. It can reduce complexity and cost by combining wireless and fiber networks, such as mobility of wireless networks and large bandwidth availability through optical networks [92, 93]. To place multiple optical units at optimal locations in FiWi, Singh and Prakash [94] used the HHO algorithm.

For many applications of wireless sensor networks (WSNs) such as intrusion detection, road traffic tracking, and oil and gas explorations, location information of the sensors is vital so that communication is not disrupted. Bhat and Venkata [95] proposed an HHO area minimization algorithm to improve the location accuracy of sensors in irregular WSN topologies. Area minimization is used in this work to minimize the search area. In a similar work, Houssein et al. [96] have used HHO to identify the ideal location for placing sink nodes in a large-scale WSN. The authors have used HHO to identify the optimal location for a sink node in WSN and used Prim's shortest path algorithm for reconstructing the WSN by choosing minimum transmission paths. In a similar work, the authors in [97] used HHO for selecting an optimal cluster head in an IoT-based network to choose the optimal routing schemes and reduce energy consumption in the IoT network. The simulation results proved the superiority of the proposed approach when compared with other recent models.

The intelligent reflecting surface is one of the techniques that can be used to provide cost-effective and green solutions to enhance the performance of WSN through the smart configuration of propagation of the signals. For example, Xu et al. [98] have employed HHO to maximize the power of the received signal by optimizing the transmit beam forming at the access point and intelligent reflecting surface's reflection coefficient.

## 5. Conclusions

In this work, we have provided a comprehensive survey on the fundamentals, variants, and applications of the HHO optimizer. Based on the existing reviews, we discovered that HHO is used in various engineering and ML applications such as clustering, classification, and feature selection. Some researchers demonstrated that HHO could efficiently solve critical optimization problems such as pattern recognition, image classification, and unconstrained optimization. At the same time, some of them provided sufficient modifications towards more harmonized exploration and exploitation trends based on the problem's nature. Furthermore, some recent works show that the hybrid variant of HHO has a faster convergence rate, optimal computational accuracy, and greater efficiency than existing metaheuristic algorithms. In our research, we discovered that HHO is efficient in all of the test problems. In the future, the work can be utilized as a guide over the recent developments on the HHO to have a better view of the current state of research on this well-known method. Also, it can be used to categorize different variants of HHO and categorize which variant is suitable for which operation, along with their advantages and disadvantages. This matter can help researchers in addressing appropriate potential problems.

## Figures and Tables

**Figure 1:** Escaping energy behavioral pattern.

**Figure 2:** Vectors during hard besiege.

**Figure 3:** Vectors during soft besiege with progressive rapid dives.

**Figure 4:** Vectors during hard besiege with progressive rapid dives in 2D.

**Figure 5:** Vectors during hard besiege with progressive rapid dives in 3D.

**Figure 6:** Input of the FHHO fuzzy inference system. (a) DF and (b) NU.

**Figure 7:** Applications of HHO.

**Algorithm 1:** HHO algorithm [8].

**Table 1:** Acronyms.

HHO	Harris Hawk optimization
AI	Artificial intelligence
SI	Swarm intelligence
PSO	Particle swarm optimization
GWO	Grey wolf optimizer
CE	Civil engineering
SCC	Soil compression coefficient
GOA	Grasshopper optimization algorithm
WOA	Whale optimization algorithm
ANN	Artificial neural networks
RMSE	Root-mean-square error
CoD	Coefficient of determination
MAE	Mean absolute error
SS	Soil slopes
HHOSA	HHO-simulated annealing
ASI	Acceleration severity index
CC	Correlation coefficient
PSO	Particle swarm optimization
GP	Genetic programming
FORM	First-order reliability method
MCE	Minimum cross-entropy
DEAHHO	Differential evolutionary adaptive HHO
MVO	Multi-verse optimization algorithm
DE	Differential evolution
SSA	Salp swarm algorithm
PSNR	Peak signal-to-noise ratio
FSI	Feature similarity index
SSI	Structural similarity index
WHHO	WAO-HHHO
CNN	Convolutional neural network
PCNN	Pulse coupled neural network
PV	Photovoltaic
TDOV	Three-diode photovoltaic
PS	Partial shading
MPPT	Maximum power point tracking
WSN	Wireless sensor networks
FiWi	Fiber wireless

**Table 2:** A summary of HHO variants.

Ref	Variant	Methodology	Objective
[19]	Multi-objective HHO	HHO is integrated with roulette wheel selection method with probability	To improve the extreme learning machine parameter selection
[20]	Gaussian barebone HHO	HHO is integrated with Gaussian barebone	To optimize kernel extreme learning machines for the prediction of entrepreneurial intention
[21]	Chaotic sequence-guided HHO	HHO is integrated with chaotic sequences	For data clustering
[22]	Dynamic HHO with mutation	HHO used mutation and dynamic control strategy to balance the exploitation and exploration phases in the HHO method	To perform segmentation on satellite and oil pollution images
[23]	Hybrid HHO differential evolution	Making two equal subpopulations from a complete one and training both the subpopulation parallelly using HHO and differential evolution	Multilevel image segmentation
[24]	Adaptive HHO	Mutation is used by HHO to clip the escape energy	Multilevel image segmentation
[25]	Hybrid OBL-HHO	OBL generates a solution for HHO through adversarial learning approach	To select the informative features from the feature space in conjunction with support vector regression
[26]	Elite OBL (EOBL)-HHO	The EOBL stacks upon OBL by selecting the fittest individual that would direct the population towards global minimum	To select informative features from the feature space
[27]	HHOBSA	The bitwise operations help HHO to improve the feature selection process, whereas the simulated annealing helps HHO to find the global minimum	Optimal feature selection
[28]	Chaotic HHO	Simulated annealing to improve HHO and the chaotic maps are used instead of random variables to achieve global optimum	To select most informative features to train using K-nearest neighbor for classification task
[13]	Salp swarm HHO	HHO is improved by adding Salp swarm optimization, which adjusts the populations and uses greedy selection to update the agent	To select the informative features
[29]	Hybrid differential evolution HHO	Nonlinear control formula balances the exploitation and the exploration of HHO throughout the convergence process	To optimize phase space reconstructions and kernel extreme learning machine parameters for wind speed forecasting
[30]	Vibrational HHO	Periodic mutations are added for enhancing swarm diversity in basic HHO method	To optimize SVM parameters for roll bearing fault diagnosis
[31]	Boosted HHO	HHO algorithm is boosted by integrating it with the exploratory phase of flower pollination algorithm and mutation step of differential evolution	To estimate the parameters efficiently for a single diode PV model
[32]	Horizontal and vertical crossover of HHO	Crisscross optimizer and the Nelder–Mead simplex algorithm are used to improve the searching capabilities of individuals for achieving faster convergence rate	Simulating an efficient PV system and extracting the unknown parameters

**Table 3:** A summary of HHO variants (continued).

Ref	Variant	Methodology	Objective
[33]	Hybrid GWO-HHO	Mutation-based GWO is used to update the bottom layer in the population, and HHO is used to find global optimal solution in the upper layer	To optimize the parameters of phase space reconstruction and kernel-based extreme ML algorithms to predict the wind speeds accurately
[34]	Modified HHO	To improve the exploration phase's global search, the Levy flight is used to generate the ambiguous zigzag position of the prey once the hawk is deducted	To relieve the PV systems from the issue of mismatch power loss problems resulting due to the phenomenon of partial shading
[35]	Chaotic HHO	HHO is enhanced with ten chaotic functions to avoid local optima trapping of conventional HHO	To accurately estimate the proton exchange membrane fuel cell's operating parameters that mimic and simulate its electrical performance
[36]	Improved HHO	Instead of random location, the rabbit location is used to find the optimal position	To find the location of distribution generation optimally in a radial distribution system to minimize the voltage deviation and total active power loss and also to increase the voltage stability index under several operational constraints
[14]	Diversification enhanced HHO (EHHO)	OBL is used in HHO to do a comprehensive search. The OBL is used to select each agent's opposite position to select the optimal agent from the available pool, and its opposite agent will be treated as the next-generation agent in HHO	To identify the optimal agents and unknown parameters of modules of PV model
[37]	Hybrid of HHO and GOA	The ensemble of GOA-ANN and HHO-ANN is performed, and then, optimal of these two is found by a process known as sensitivity analysis	To optimize the artificial neural network for predicting SCC dataset
[38]	HHOSA	SA is used to optimize HHO and improve its global convergence	To optimize the design parameters of highway guardrail systems
[39]	HHO-FORM	The reliability index is formulated in the HHO-FORM model for a constrained optimization problem. Later, the exterior penalty methodology is used to handle the constraints. HHO determines the optimal reliability index to improve the convergence through the strategy of Levy Flight and population-based mechanism	To reduce the high dimensionality in designing and analyzing risks of structuring in civil engineering
[40]	HHO-minimum cross-entropy (MCE)-MCET-HHO	MCET is used as a fitness function in HHO for determining optimal thresholds to segment an image	To find the optimal configuration of thresholds for image processing
[41]	Hybrid WHHO	WOA is integrated with HHO to improve the convergence rate of HHO in obtaining global optimum	To classify brain tumor using MRI images

**Table 4:** A summary of HHO variants (continued).

Ref	Variant	Methodology	Objective
[42]	Differential evolutionary adaptive HHO	The HHO is updated by making the Harris Hawk adaptive to decide when it has to move to a random tall tree or when it has to do perching. Also, to improve the exploration ability of HHO, the authors have used the differential evolutionary concept	To improve the exploration ability of HHO for multilevel image thresholding
[43]	Hybrid HHO-SSA	To overcome the HHO's property of stagnating in local optima and prevent immature convergence during exploitation and exploration. The initial solutions generated are divided into two halves in which HHO's exploratory and exploitation are applied to the first half, and SSA's searching stages are utilized to update solutions in the other half. Hence, HHO-SSA chooses the best solution among the two	To address the global optimization problem and find the optimal threshold values
[44]	Hybrid multi-population differential evolution-HHO	The exploitation phase of the HHO is enhanced by chaos. The multi-population strategy is used to improve the ability of global search. Later, differential evolution is used to improve the quality of the solution from the previous stage	To optimize de-noising in satellite images in wavelet domain
[23]	HHO and differential evolution (DE)	Kapur's entropy and Otsu's method are used as fitness functions to find the threshold values of segmentation. The proposed model divides the entire population into two equal parts assigned to DE and HHO algorithms. During the iterative process, both HHO and DE will update each subpopulation position simultaneously	To extract optimal features from images for segmentation of color images, the optimal threshold values of segmentation are found
[22]	Dynamic HHO with mutation	HHO is integrated with a novel dynamic control parameter strategy to avoid the HHO being trapped in the local optimum. A disturbance term is added to update the formulation of the escaping energy formulation. Cosine and sine are integrated to control when the disturbance peak appears. To increase the randomness of the HHO, a Gaussian distribution is adopted	To segment the satellite images
[45]	Hybrid cuckoo search-HHO	To strengthen the HHOs being trapped in local solutions, inaccuracy, inadequate search coverage, and slow convergence, cuckoo search's property of dimension decision strategy, and Gaussian mutation are integrated with the HHO during exploration and exploitation phases	To optimize the parameters in cantilever beam design problem, welded beam design problem, and tension/compression spring design problem
[46]	Hybrid HHO-SSA	SSA is employed to enhance the performance of HHO by acting as a local search for HHO	To enhance the performance of HHO by acting as a local search for HHO
[47]	Hybrid HHO-WOA	HHO is applied to the first half of the population, and WOA is applied to the second half. Hence by integrating WOA with HHO, the exploitation and exploration phases of HHO are enhanced to select the optimal parameters	To predict the values of several parameters such as hydrocarbon, brake thermal efficiency, carbon monoxide, and carbon dioxide based on the data gathered from the experimental setup of the dual-fuel engine by varying injection timings, blends of rice bran biodiesel, engine operating load, and air-fuel ratio

## Data Availability

No data are used in this work.
